# Involvement of GABA_A_ Receptors in the Anxiolytic-Like Effect of Hydroxycitronellal

**DOI:** 10.1155/2021/9929805

**Published:** 2021-06-16

**Authors:** Jéssica C. Andrade, Álefe B. Monteiro, Humberto H. N. Andrade, Thallita K. S. N. Gonzaga, Pablo R. Silva, Danielle N. Alves, Ricardo D. Castro, Mayara S. Maia, Marcus T. Scotti, Damião P. Sousa, Reinaldo N. Almeida

**Affiliations:** ^1^Psychopharmacology Laboratory, Institute of Drugs and Medicines Research, Federal University of Paraíba, Campus I, 58051-085, Via Ipê Amarelo/SN, João Pessoa, Paraíba, Brazil; ^2^Department of Clinic and Social Dentistry, Center for Health Sciences, Federal University of Paraiba, Campus I, João Pessoa, PB, Brazil; ^3^Cheminformatics Laboratory, Institute of Drugs and Medicines Research, Federal University of Paraíba, Campus I, 58051-900, Via Ipê Amarelo/SN, João Pessoa, Paraíba, Brazil; ^4^Pharmaceutical Chemistry Laboratory, Institute of Drugs and Medicines Research, Federal University of Paraíba, João Pessoa, Brazil

## Abstract

Hydroxycitronellal (HC) is a monoterpene present in essential oils of aromatic plants of different species, obtained from semisynthesis of citronellal, and is widely used as a fragrance in cosmetics. The objective of this work was to evaluate the possible anxiolytic-like activity of HC and its possible mechanism of action using *in vivo* and *in silico* methodologies. Swiss male mice (*Mus musculus*) were treated with HC (12.5, 25, and 50 mg/kg, i.p.) and subjected to the rota rod, elevated plus maze, and open field tests. No significant impairments were observed in the rota rod tests for the motor activity of the animals treated with HC at 12.5, 25, and 50 mg/kg, i.p., indicating no myo-relaxing or sedative effects. In the elevated plus maze, HC (in the three doses) induced significant increases in the percentage of entries (respectively, 34.8%, 33.8%, and 38.6%) and in the length of stay (respectively, 49.9%, 56.1%, and 57.0%) in the open arms of the EPM, as well as the number of crossings in the open field tests. The mechanism of action of the compound's anxiolytic-like activity can be attributed to the involvement of GABA_A_ receptors, and this interaction was observed in *in vivo* and *in silico* studies. For HC, the results suggest anxiolytic-like effects, possibly via modulation of the GABAergic system. The use of natural products to treat anxiety can become an alternative to existing synthetic products.

## 1. Introduction

Anxious behavior is part of the normal spectrum of human experience. In certain situations, all people in life experience anxiety, especially when faced with some warning of imminent danger. This reaction allows us to escape from dangerous situations, as well as to improve our response in the face of adverse conditions when imposed by the environment [1]. If the risk response is emotionally disproportionate to the situation that triggers it, anxiety becomes a disorder [2].

Inherited genetic, neurobiological, environmental, and traumatic experiences can trigger pathologically anxious behavior. Anxious disorders are a clinical condition in which anxiety is the primary symptom and does not originate in other disorders, such as depression [3]. According to the World Health Organization, the proportion of the population who present some type of anxiety disorder in the world is 3.6%, that is, 256 million people, being more common in women (4.6%) than in men (2.6%) [4].

Pathological anxiety is treated with anxiolytic agents, which are substances that act on the central nervous system (CNS), resulting in changes in behavior, perception, thoughts, and emotions. They are recommended for people who suffer from emotional and psychological disorders that affect the functioning of the mind [5].

Benzodiazepines (BZDs) are a class of substances presenting anxiolytic effects and, due to their wide therapeutic window, high therapeutic efficacy. These drugs act through GABA_A_ ionotropic receptors, intensifying inhibitory neurotransmission. Clinically, diazepam (DZP) is one of the most frequently used BZDs, and (similar to other BZDs) sedation is one of its more evident adverse reactions; it directly affects locomotor activity and compromises the quality of life of the user [6, 7].

Alternatives are needed to develop anxiolytics which possess fewer adverse reactions, possibly using medicinal plants, since they are an excellent source of bioactive substances which can present a great influence on health [8]. Medicinal plants with psychoactive activity present important effects on consciousness, emotions, and cognition, and due to these effects, they are used for many purposes. Pharmacological studies involving medicinal plants, especially aromatic ones, which present activity on the CNS, have helped to promote our understanding of the neurochemical base of behavioral disorders, making it a favorable field for the development of new drugs [9, 10].

Essential oils (EO) are odorous substances [11]. Formed in plant secondary metabolism, they act as a form of protection against predatory attacks, to attract pollinators, and have many other activities. The great structural variety of substances present in EOs is one of the factors responsible for their various pharmacological activities, including anxiolytic [12], antidepressant [13], anticonvulsant [14, 15], and antinociceptive effects [16–20]. Some of these activities are attributed to the intensification of GABAergic transmission due the interaction of monoterpenes with GABA_A_ receptors [21].

Hydroxycitronellal (HC) is a monoterpene present in essential oils of the most diverse genera of aromatic plants, yet little reported in the literature regarding its pharmacological effects. This monoterpene can be obtained from another monoterpene and citronellal, a metabolite of plant origin that already has several pharmacological activities proven in the literature, such as analgesic [22], anxiolytic [23], and anticonvulsant [24] activities. In view of the promising activity of one of its precursors (citronellal) in the CNS, the present study is aimed at evaluating the anxiolytic effect of HC and evidence of modulation of the GABA_A_ receptor with acute administration in vivo and in in silico trials.

## 2. Materials and Methods

### 2.1. Animals

Swiss mice (*Mus musculus*), albino adult male, weighing between 25 and 35 g, approximately 3 months old, kept under temperature control (21 ± 1°C), with free access to water and feed, and a 12-hour light/dark cycle were used for all experimental protocols. The animals came from the Animal Production Unit (APU) of the Pharmaceuticals and Medicines Research Institute (IPeFarm) of the Federal University of Paraíba. All experimental procedures were previously approved by the CEUA-Ethics Committee on the Use of Animals at UFPB, under the certificate No. 1854110719.

### 2.2. Drugs

HC was purchased from Sigma-Aldrich® ChemicalCo (St. Louis, MO, USA). Diazepam and flumazenil were donated by the Brazilian pharmaceutical laboratory, Cristália-Produtos Químicos Farmacêuticos, LTDA (Itapira, SP, BR). All substances were diluted in saline and intraperitoneally administered (i.p.) at a total volume of 0.1 mL/10 g. HC was initially emulsified with Tween 80 (0.5%) in 0.9% saline. The control group received the vehicle (Tween 80-0.5% in 0.9% saline).

### 2.3. *In Vivo* Testing

#### 2.3.1. Estimate of Acute Toxicity of Hydroxycitronellal

The acute toxicity tests were performed according to the OECD “Guidelines for testing of chemicals” n. 423/2001with modifications. Swiss mice, three females per group, including the control, were subjected to single doses of 2000 and 300 mg/kg of HC. The control group was treated with 0.9%saline + 5%Tween intraperitoneally. After administration, observations were made at 30 min, 1 h, 2 h, and 4 h and then once daily until the fourteenth day.

#### 2.3.2. Rota Rod

The rota rod methodology assesses motor impairment in animals after administration of substances with potential CNS activity. The animals were exposed to the apparatus 24 h before the test, and the animals managing to stay on the rotating bar (at 10 rpm) for a period of 1 minute were selected for testing. These preselected animals (*n* = 8) were treated (i.p.) with vehicle (control group: Tween 80-0.5%), diazepam (4 mg/kg), administered 30 min before the start of the test, or HC (12.5, 25, and 50 mg/kg). At 30, 60, and 120 minutes, the animals were placed on the rotating bar to assess time performance. For each animal, the time spent on the rotating bar was recorded for 3 minutes [25, 26]. The doses of HC were defined from the acute toxicity study and previous studies [27, 28].

#### 2.3.3. Elevated Plus Maze Test

Groups of mice were used (*n* = 8). Substances, vehicle (control group: Tween 80-0.5%), diazepam (1 mg/kg), or HC (12.5, 25, and 50 mg/kg) were administered 30 min before the start of the test, intraperitoneally. After 30 minutes, each animal was placed individually on the central platform of the device, facing an open arm. The observed behavioral parameters were the number of entries and length of stay (in seconds) in the open arms and closed. An entry was counted only if the animal had four legs outside of the central line of the labyrinth. Each animal remained for a time of 5 min in the maze [29].

#### 2.3.4. Open Field Test

The animals were submitted to the open field test and evaluated for a period of 5 minutes. For the experimental procedure, groups of 8 mice were used. HC (12.5, 25, 50 mg/kg), vehicle (control group: Tween 80-0.5%), and diazepam (1 mg/kg) were administered intraperitoneally, 30 min before the start of the test. After treatment (30 minutes), each animal was individually submitted to the device. The total number of quadrants covered (crossings), head rearing, and time spent on grooming was recorded [30].

#### 2.3.5. Involvement of GABAergic Receptors in Anxiolytic Activity

This test was carried out with the aim of evaluating the possible involvement of GABA_A_ receptors in the anxiolytic effect of the substance. The animals were divided into three pretreated groups (*n* = 8), vehicle (control group: Tween 80-0.5%), diazepam (1 mg/kg), and HC (12.5 mg/kg), 30 min before the start of the test. 20 min before starting treatments, all groups were pretreated with flumazenil (10 mg/kg), a GABA_A_ receptor antagonist. Then, the animals were submitted to the elevated plus maze test. The observed behavioral parameters were number of entries and length of stay (in seconds) in the open arms. An entrance was counted only if the animal had four legs in one of the two open arms of the labyrinth [31].

### 2.4. *In Silico* Testing

#### 2.4.1. Docking Consensus

The HC structure was obtained in (.sdf) format through ChemAxom (http://www.chemaxon.com). The *α* subunit of the GABA_A_ receptor, under the code PDB ID 6HUJ, was obtained from the Protein Data Bank (PDB) (http://www.rcsb.org/). The ChemAxon (http://www.chemaxon.com) Standardizer Software JChem 14.9.1.0, 2014, was used to expose the HC structure, add hydrogens, perform aromatic shape conversion, outline the molecular graph in 3D, and generate compounds in the .sdf format [32].

Docking was performed using five different scoring functions (Molegro Virtual Docker (MVD), Gold 5.6.2, AutoDockVina (Vina), AutoDock 4.2.6. (AD4), and Plants). The water molecules were removed from the crystalline structure, and the mean square root deviation (from the “Root Mean Square Deviation” (RMSD)) of the poses was calculated, indicating the degree of docking reliability. The consensus strategy consisted of selecting predicted binding affinity values greater than the crystallographic ligands in at least three docking programs. The results were viewed using the Molegro Virtual Docker v.6.0.1 (MVD) software [33] and the Discovery Studio 2019 (https://www.3dsbiovia.com/products/collaborative-science/biovia-discovery -studio/visualization-download.php).

#### 2.4.2. Molecular Dynamics Simulations

The GROMACS 5.0 software was used to perform molecular dynamics simulations [34]. Ligand topology was prepared using the ATB topology generator (https://atb.uq.edu.au/) [35, 36] and applying the GROMOS96 54a7 force field. Protein topology was also prepared using the GROMOS96 54a7 force field in GROMACS. Molecular dynamics simulation was performed using the SPC water model with a point charge in a cubic box [37]. The system was neutralized with the addition of ions (Cl^−^ and Na^+^) and balanced at 300 K using the V-rescale algorithm at 100 ps, represented by NVT (constant number of particles, volume, and temperature), followed by equilibrium at 1 atm pressure using the Parrinello-Rahman algorithm-NPT (constant number of particles, pressure, and temperature) up to 100 ps. The MD simulations were performed in 5,000,000 steps at 10 ns. The mean square root displacement (RMSD) of all C*α* atoms was calculated in relation to the starting structures. Residual fluctuations (RMSF) were also analyzed to understand the role of residues near the receptor binding site. The RMSD and RMSF graphs were generated in the Grace software (http://plasma-gate.weizmann.ac.il/Grace/), and the protein and ligands were visualized in UCSF Chimera [38].

#### 2.4.3. Pharmacokinetic Predictions

Pharmacokinetic predictions (available for free) were obtained from electronic platforms: SwissADME (Swiss Institute of Bioinformatics, Switzerland) and Xenosite (Washington University of Medicine, United States). For predictive models interfacing, it was necessary that the structures were in the smile format, being generated by the Chemdraw Ultra 12.0 software [39].

#### 2.4.4. Statistical Analysis

The results obtained in the *in vivo* experiments were analyzed using the software and one-way analysis of variance (ANOVA), followed by the Tukey test to compare the means. Data were expressed as mean ± S.E.M. (standard error of the mean), and a confidence level of 5% was adopted.

## 3. Results

### 3.1. *In Vivo* Testing

#### 3.1.1. Estimate of Acute Toxicity of Hydroxycitronellal

With administration of HC at a dose of 2000 mg/kg, i.p., all animals died, making it necessary to decrease the dosage, as determined by the OECD (2001). HC was then administered at a dose of 300 mg/kg, i.p., and did not cause the animals to die. In view of the results, it was the estimated LD50 of the tested substance (HC) at 500 mg/kg. Using this result, to conduct pharmacological tests *in vivo*, we opted for HC in doses 12.5, 25, and 50 mg/kg, since doses below the LD_50_ value present a lower probability of being toxic.

#### 3.1.2. Rota Rod

After administration of HC (i.p.) at doses of 12.5, 25, and 50 mg/kg, there were no significant differences in the length of stay of the animals on the rotating bar (tested after 30, 60, and 120 minutes) in relation to the control group (Figure 1). The animals in the DZP group did not remain on the rotating bar at the evaluated times.

#### 3.1.3. Elevated Plus Maze Test

The results presented in Figure 2(a) demonstrate that the animals treated with HC at 12.5 (6.6 ± 0.3), 25 (6.5 ± 0.5), and 50 (7.0 ± 0.3) mg/kg significantly increased the number of entries into the open arms of the labyrinth, in relation to the control group (4.3 ± 1.0), by 34.8%, 33.8%, and 38.6%, respectively. The diazepam-treated group also significantly increased the number of entries (63.5%) compared to the control.

The results obtained for the animals' permanence in the open arms are shown in Figure 2(b). HC at the dose of 12.5 (89.8 ± 2.7), 25 (102.7 ± 9.8), and 50 (104.5 ± 6.3) mg/kg significantly increased the animals' permanence time in the open arms of the labyrinth, respectively, by 50.0%, 56.1%, and 57.0% compared to the control group (45 ± 2.6). The diazepam administered group (152.3 ± 5.0) also presented significant results, increasing the animals' permanence in the open arms of the device by 70.4% compared to the control group.

Figure 2(c) shows the results of the number of entries, of the animals, in the closed arms of the labyrinth. The animals treated with HC at doses of 12.5 (4.5 ± 0.7), 25 (5.3 ± 0.8), and 50 (4.7 ± 0.9) showed significant differences when compared to the control group (12.0 ± 1.0); that is, the animals entered less into the closed arms of the labyrinth. The group treated with DZP also showed significant results, with a decrease in the number of entries in the closed arms (2.2 ± 0.4).

As for the length of stay in the closed arms, the animals treated with HC at doses of 12.5 (137.5 ± 17.6), 25 (163.0 ± 7.3), and 50 (170.1 ± 17.6) exhibited significant differences when compared to the control group (247.5 ± 16.0); that is, the animals spent less time in the closed arms of the labyrinth. The group treated with DZP also showed significant results, with a decrease in the number of entries in the closed arms (2.2 ± 0.4).

#### 3.1.4. Open Field Test

As to the animal ambulation behavior in the open field tests, the results are shown in Figure 3(a), and it was noticed that there was a significant increase in the movement of animals treated with HC at 12.5 (83.8 ± 4.0), 25 (82.0 ± 10.6), and 50 (71.0 ± 7.6) mg/kg, respectively, by 71.5%, 71.0%, and 66.5% compared to the control group (23.8 ± 1.5). The DZP group (74.2 ± 1.5) increased the animals' ambulation by 67.9% when compared to the control group.

Figure 3(b) presents the results obtained for rearing. It can be observed that the HC groups at 12.5 (25.8% ± 2.9), 25 (19.1 ± 2.5), and 50 (14.0 ± 2.9) mg/kg expressed a significant increase in head rearing behavior of 89.5%, 85.8%, and 80.7%, respectively, when compared to the control group (2.6 ± 0.4). The DZP group (16.4 ± 1.5) increased this same behavior by 83.4%.

The results obtained for the grooming parameter can be seen in Figure 3(c). It is noticed that there was a significant difference in grooming time only in the group treated with HC at a dose of 25 mg/kg (60.3 ± 13.6), decreasing by 50.1% in relation to the control group (121.1 ± 13.1). In the group treated with DZP (1.2 ± 0.2), the decrease was 99.0%. The other doses of HC presented no significant differences in relation to the control group.

#### 3.1.5. Effect of GABAergic Neuromodulation on the Anxiolytic Effects of HC

The results of Figure 4(a) (number of entries in the open arms of the EPM) reveal that the flumazenil + HC 12.5 group (4.1 ± 0.5) presented a lower number of entries, at 12.7%, less than presented by HC (at 34.8%), and at a dose of 12.5%, when administered without the antagonist. The antagonist when administered with DZP (4.3 ± 0.4) also reduced the number of entries to the open arms, yielding a percentage of 8.5%, which was less than that presented when DZP was administered alone (11.8 ± 0.2), at 63.5%. These results were not significant when compared to the control group (4.7% ± 0.4).

Figure 4(b) presents the results for the time spent by animals in the open arms of the EPM. The animals in the group treated with HC at 12.5% presented a permanence time of 49.9% (89.9 ± 2.7), this falling to 25.3% (35.3 ± 4.3), after pretreatment with the antagonist. The same occurred with DZP, which saw its percentage of permanence time fall from 70.4% (152.3 ± 5.0) to 6.5% (50.6 ± 5.6) after administration of flumazenil, with no significant differences when compared to the control group (47.3 ± 3.4).

### 3.2. *In Silico* Testing

#### 3.2.1. Docking Consensus

In this study, the results generated using the five scoring functions were validated through redocking of the crystallographic ligand. The RMSD of the positions obtained was calculated. Redocking consists of positioning and predicting the binding affinity of the crystallographic ligand in the region of the active site receiver. The RMSD compares and calculates the mean square root deviation of the positions obtained by redocking, and the ligand structure obtained experimentally. For docking to be considered reliable, the RMSD value must be equal to or less than 2.0 Å.

The programs MVD, Vina, and AD4 select the best binders for the most negative energy values, while the Gold and Plant programs select the best binders for the most positive energy values. HC obtained a higher binding affinity value than the crystallographic ligand (ABU), a cryo-EM structure of the *α*1*β*3*γ*2L receptor subunits in complex with GABA, in at least three of the programs (Table 1), indicating a satisfactory degree of affinity for the GABA_A_R. Computational techniques were then used to assess the stability of the bond.

Figure 5 reveals that HC managed to form more stable interactions through hydrogen bonds with residues Arg67, Thr202, and Tyr157 in the region of the active site, whereas the ABU ligand formed a hydrogen interaction only with the amino acid Ser156. Steric interactions were also observed between residues Tyr205 and Tyr97 and the HC ligand, as well as interactions over short distances, which are more stable with residues Arg67, Tyr157, Thr202 and Tyr205, and HC.

#### 3.2.2. Molecular Dynamics Simulations

The molecular dynamics (MD) simulations were performed taking into account the best results obtained in the consensus docking. The interactions between GABA_A_R and HC were evaluated, and the crystallographic ligand (ABU) was used to study the flexibility and conformational changes in the complexes during the MD simulations. For this, the mean quadratic deviation (RMSD) was separately calculated for the C*α* atoms of the protein and the structures of each ligand. The RMSD analysis of GABA_A_R revealed that the protein reached conformations ranging from 0.3 to 0.4 nm in size in 10 ns. The results demonstrated that the protein is stable (Figure 6(a)), presenting no significant changes. In addition, when comparing the flexibility of the complexed protein to the ligands, we found that HC complexed to GABA_A_R remained stable most of the time, while the crystallographic ligand (ABU) complexed to GABA_A_R revealed structural change peaks between 3 and 4 nm.

RMSD analysis of the ligands revealed that HC is more stable than ABU (Figure 6(b)), suggesting that, although the protein undergoes minor structural changes, HC tends to remain within the active site longer, and the binding affinity is not lost, even in the presence of different factors such as temperature, solvent pressure, and ions.

To understand the flexibility of the residues and amino acids that contribute to GABA_A_R conformational changes, the mean square root fluctuation (RMSF) of each receptor amino acid was calculated. Residues with higher RMSF values suggest greater flexibility, while low RMSF values suggest less flexibility. Considering that amino acids with fluctuations above 0.3 nm contribute to the flexibility of the protein structure, we found that of the E and D chain amino acids that interacted with the agonist ligand ABU, not one contributed to a conformational change in the protein (Figure 6(c)). Since the active site is stable, the binding affinity for the compound tends to remain unchanged.

The docking interactions observed for the GABA_A_R-HC complex were stable during the molecular dynamics simulations. When analyzed using graphics programs, it was noted that HC loses interactions with the amino acids observed in docking (Figure 7), suggesting new interactions, appearing mainly through hydrogen bonds with the amino acids Phe35, Phe54, Arg56, and Glu492. Various factors may have contributed to this exchange of interactions between amino acids, such as for example, the interaction with compounds presenting water molecules and ions within the system defining the molecular dynamics.

#### 3.2.3. *In Silico* Pharmacokinetic Predictions

The properties of medicines obtained in the ADMET system are the principal characteristics evaluated during the development phase of a future medicine. In new drug development, the ADMET forecast provides guidance that minimizes failure rates [40].

*In silico* pharmacokinetic predictions (Table 2) were performed using the ADMET parameters, with the aim of identifying possible pharmacokinetic disadvantages in the HC substance. According to Lipinski's rules, a potential drug is orally active when it meets the following criteria: (a) molecular weight ≤ 500 Da, (b) Log*P* ≤ 5 (or MLog*P* ≤ 4.15), (c) number of hydrogen bond acceptors ≤ 10, and (d) number of hydrogen bond donors ≤ 5 [41].

HC presented a Log*P* of 2.15, as well as adequate number of donors and acceptors of hydrogen bonds, complying with Lipinski rules and suggesting good bioavailability. In relation to Log*S*, the value found for the compound was in the appropriate range (-4 and -2), indicating adequate solubility, which directly favors the bioavailability of the compound [42].

Molecules that present TPSA (Topological Polar Surface Area) values of less than 140 Å^2^ and values above 0.90 (log Papp; log cm/s), for the Caco-2 parameter, suggest that the substance presents a good profile for intestinal absorption. Such *in vitro* models are widely used to assess these parameters [43].

The volume of distribution (VDss) indicates the theoretical volume of a given substance evenly distributed in the blood plasma. Values below 0.45 (log L/kg) indicate a good plasma distribution, with the substance being readily available to interact with its biological target. Elimination of the substance did not increase because of its free form, as was observed for renal clearance (clearance/mL/min/kg). The greater the total clearance, the greater and faster the elimination of the substance will be [42, 44].

## 4. Discussion

According to a preliminary study, the oral LD50 of 7-HC was 5000 mg/kg [45]. In view of this result, the study of the LD_50_ estimate was initiated using the dose of 2000 mg/kg, i.p., aiming not to reach the lethal dose previously stipulated. However, even with the dose reduction to 2000 mg/kg, all animals died. This may have been due to the route of administration used. Therefore, the dose was again decreased, this time to 300 mg/kg.

In the initial toxicity test, during the 14-day observation period, after the administration of 300 mg/kg, i.p., no changes were found that would indicate toxicity, such as changes in the skin, hair, eyes, or respiratory system. The data demonstrated that under the evaluated conditions, HC presents low toxicity, providing an incentive to conduct *in vivo* pharmacological tests and allowing the choice of safe doses for these tests [9].

*In vivo* methodologies assess the anxiolytic-like activity of substances by inducing inhibitory behaviors in animals, in contrary to the stress caused by the environment to which they are subjected [46]. These inhibitory behaviors can be expressed by not realizing a movement or by increasing permanence time; these, since naturally, rodents are natural explorers. Substances with potential anxiolytic action must be able to reduce these inhibitory behaviors [47].

The behavioral changes induced upon HC administration (i.p.) were evaluated using the rotating bar (rota rod), elevated plus maze, and open field tests; these tests are well established in the study of substances with central nervous system activity, and except for the rotating bar test, they are models based on the observation of innate animal behavior, that is, on the ethology of rodents.

Rota rod testing is a classic animal model used to assess the influence of unknown substances on an animal's motor coordination [26] when affected by agents such as benzodiazepines and anesthetics [25]. The test is carried out to illustrate the possible interference of the administered substance on motor coordination. Diazepam (DZP) causes impairment of balance or motor coordination, possibly due to neurotoxicity and thus restricts patient quality of life [48]; the use of diazepam (DZP), a reference drug in the treatment of anxiety (responsible for most reported side effects), as a control, allows comparison of motor locomotion impairment upon administration of HC. As was observed in the rota rod test, the animals' locomotion was not compromised with administration of HC, differently from what was seen in the group treated with DZP. Thus, HC did not compromise the animals' motor coordination.

To better evaluate the possible HC anxiolytic effects, the animals were subjected to the EPM test, which is considered one of the most well-established tests and the reference standard for detecting anxiolytic and anxiogenic effects [49]. The EPM test induces a conflict in the animal between exploring new environments and the tendency to avoid dangerous areas [47]. The administration of HC, in the three studied doses, significantly increased the percentage of entries and permanence in the open arms of the apparatus, in relation to the control group, indicating that acute administration of the compound increased the exploration behavior in the apparatus, indicating possible anxiolytic activity. The results are in line with studies that have demonstrated the anxiolytic activity of volatile, monoterpenoids, such as limonene, linalool, citronellal, and geranial, using the EPM methodology [46, 50, 51].

The open field test is widely used to assess behavioral effects of compound administration, especially in locomotor and anxious parameters [52, 53]. HC in the three doses tested was able to increase the locomotion of the animals towards exploring the apparatus quadrants, mainly the central quadrants. This behavior is associated with decreased anxiety levels in the animals, even when submitted to a new and stressful environment. In addition to the total number of crossings, other parameters can be observed in the open field test, such as the amount of self-cleaning (grooming) and vertical surveys (head rearings) [54, 55]. Thus, the greater the anxiety, the less number of head rearings and the more grooming. After treatments, the head rearing values increased significantly for the doses of 12.5 and 25 mg/kg, compared to the control group. The amount of grooming activity was reduced only when the dose of 25 mg/kg was administered. Reduction in self-cleaning is often seen in animals treated with compounds with potential anxiolytic activity [56]. The increase in the number of crosses in the open field test can be corroborated with the increase in the number of entries in the open arms of the elevated plus maze. The HC did not cause any change in the animals' locomotion; this is proven due to the greater safety of the animals in walking through these regions of the labyrinth. The number of entries and length of stay, decreased, in the closed regions of the device, also reinforces this idea.

Finally, to assess whether the effects observed with HC involve interaction with the GABAergic system, the benzodiazepine GABA_A_ receptor antagonist flumazenil was used. The antagonist was administered before the substances under study. If the pharmacological effect was reversed or even decreased significantly, it would mean that the antagonist, when binding to the target, prevented the substance from binding, and consequently, the pathway was involved in the pharmacological effect [57].

Pretreatment with the antagonist flumazenil reversed the anxiolytic-like effect of HC, as well as DZP, suggesting that HC is capable of reducing anxiety through a mechanism of action similar to that of BZDs (GABA_A_R). Interactions between GABA_A_R and other essential oils as well as their isolated compounds, such as citronellal, have been shown to result in CNS depressant activity [58–60].

The positive modulation of the GABA_A_ receptor by the enantiomer of the bicyclic monoterpene borneol, found in essential oils of medicinal herbs, such as valerian, was observed using electrophysiology models. Borneol directly activated GABA_A_ receptors, producing 89% and 84%, respectively, of the maximum GABA response indicative of a partial agonist action, being insensitive to flumazenil, indicating that (+)- and (-)-borneol did not act in the classic sites of benzodiazepines [61]. HC has been shown to interact with the GABAA receptor in a common place for benzodiazepine binding, as its effect has been reversed by flumazenil. However, both studies demonstrate the interaction of these substances with the GABAergic receptor.

As discussed by Jiménez-Ferrer et al. [62], evaluating the anxiolytic effects of *Aloysia triphylla* fractions, which contained 21.6% citronellal, employed the EPM test and concluded that all fractions studied induced an anxiolytic-like effect. The activity was reversed with the use of a flumazenil antagonist. In another study, the sedative properties of *Melissa officinalis* include stress, agitation, and anxiety reduction which are attributed to the presence of phytochemicals, including citronellal (2.92%). The anxiolytic activity of *M. officinalis* has been attributed to a possible interaction with GABA_A_ receptors, assuming activity similar to that of BZDs [63].

According to the position of Santos et al. [27], testing citronellal complexed with *β*-cyclodextrin observed an increase in the neuronal excitation threshold and a resulting decrease in muscle hyperalgesia. This effect is probably due to CNS activation, as discussed by Melo et al. [64] using the hot plate test, which had previously demonstrated that citronellal presents a central analgesic effect probably due to interaction with the GABA_A_R.

Substances that bind to GABA_A_R, such as benzodiazepines, cause a change in the conformational state of the receptor, which promotes increased affinity for the GABA neurotransmitter, stimulating the opening of GABA_A_R channels [65]. This results in hyperpolarization of the cell, reduced neuronal activity, and modified emotional states, all through anxiolytic, sedative, and muscle relaxing actions.

According to the data, the interaction of HC with GABAAR can result in greater neuronal hyperpolarization. After HC-GABAAR receptor binding, a greater influx of Cl- into the cell is suggested, regardless of GABA binding. Accumulation of chloride ions inside of the cell increases the threshold of neuronal excitation and prevents nerve impulse conduction [60, 66]. This general decrease in excitation can act in relieving the characteristic symptoms of anxiety.

Using *in silico* methodologies, the possible anxiolytic activity of the compound was also evaluated through involvement of the GABA_A_ receptor, a principal biological target for anxiolytic substances. Computational methodologies, used in the initial stages of drug development, can unveil the character of unknown molecules and evaluate potential biological targets to better direct further study [67]. The most important inhibitory neurotransmitter in the central nervous system, without doubt, is gamma-aminobutyric acid (GABA). Any factor that promotes decreases in GABAergic transmission will result in the triggering of anxious and aggressive behaviors [68]. Through knowledge of the hydroxycitronellal (HC) structure, as well as that of GABA_A_R, it was possible to identify the potential agonist activity of the compound for this receptor, this, through the process of molecular complementarity [69].

When compared with the amino acids involved in the BZD-GABA_A_R interaction, the interaction of HC with GABA_A_R (through different amino acids) may be responsible for the observed nonimpairment of the test animals' motor coordination. This revealed the potential of HC for use in formulating a new anxiolytic medication, which might allow patients to perform their daily functions normally, without the risk of accidents.

The hydrogen interactions between the amino acid residues of GABA_A_R and HC, compared to the ABU crystallographic ligand, presented greater affinity. The interactions between an enzyme and its substrate are complementary and were initially introduced in the famous “key-lock” model, proposed by Fischer [70]. Such complementarity, at the molecular level, would be observed through intermolecular interactions, represented by hydrophobic interactions, van der Waals, *π* clouds, hydrogen bonds, and electrostatic interactions [71].

Previous molecular docking studies between diazepam (DZP) and GABA_A_Rs [72] indicate that the drug binds to amino acids Lys105, Tyr160, Tyr210, and Val212 in the *α*1 subunit and to the amino acid Phe77 in the *β*2 subunit. HC in its stable binding form interacted with Arg67, Thr157, and Tyr157; this difference in amino acid binding is potentially the reason that the interaction between HC and GABA_A_R is more stable.

Molecular dynamics is important since it assesses structural differences between molecules, as was done for the HC and ABU agonists. The higher the RMSD value, the greater the structural difference between the proteins or structures were compared, as was observed for the HC ligand [73].

In this study, low RMSD values (>0.3 nm) were observed for the majority of the simulation time, indicating greater HC stability in the system compared to the crystallographic ligand (ABU). Sudden changes in RMSD denote important conformational changes in the molecule, while small RMSD oscillations indicate system equilibrium [74]; the equilibrium directly influences the interaction of the ligand and its receptor.

Through the molecular dynamics (MD) results, more stable HC-GABA_A_R bonding was observed. This stability may be related to the hydrogens of the CHO (aldehyde) functional groups, which can participate in nonclassical hydrogen bonds with certain amino acid residues, and such interactions with GABA_A_R amino acids can result in chloride ion influx into the cell, decreasing neuronal excitation.

To establish an adequate pharmacokinetic profile for HC, absorption, distribution, metabolism, excretion, and toxicity (ADMET) parameters were also evaluated. Absorption and distribution directly influence the bioavailability of the substance, while metabolism and excretion affect the rate of elimination of the substance from the body. Proper disposal of substances decreases the chances of toxic events being triggered [43].

To present a good bioavailability, a drug must obey at least three of the following parameters: molecular weight less than or equal to 500 Daltons (Da), high lipophilicity (Log*P* of less than 5), number of hydrogen bond donors (HBD) less than 5, and number of hydrogen bond acceptors (HBA) less than 10 [41]; no violation of these parameters was observed for HC.

HC was administered intraperitoneally in *in vivo* experiments, mainly due to its physical-chemical characteristics, such as liposolubility. The liposolubility of a substance determines its ability to permeate biological membranes and to reach its target [75]. The pharmacokinetic predictions revealed that HC has sufficient lipophilicity to interact with the lipid bilayer of biological membranes, as well as a water solubility compatible with the dissolution of the molecule in the aqueous biological fluid, resulting in good absorption.

## 5. Conclusions

Based on the data obtained in the present work, it is possible to conclude that hydroxycitronellal presents anxiolytic-like effect, which likely occurs through positive modulation of GABA_A_ receptors. Ruling out HC neurotoxicity, the compound's anxiolytic-like activity did not present adverse effects, such as sedation and neuromuscular impairment commonly observed in benzodiazepines. These findings reinforce the pharmacological potential of the monoterpene citronellal and its derivatives, such as hydroxycitronellal.

## Figures and Tables

**Figure 1:** Effect of HC (mg/kg, i.p.), the time of stay (s) of the animals on the rota rod. The column represents the average ± S.E.M. (*n* = 8). Statistical analysis: ANOVA unidirectional (*F* value = 177.4) followed by the Tukey test, ^∗^*p* < 0.05, ^∗∗^*p* < 0.01, ^∗∗∗∗^*p* < 0.001: (HC) = vs.control and (DZP) = vs.control.

**Figure 2:** Effect of HC (mg/kg, i.p.) and diazepam, number of entries (a) (*F* value = 42.3), the time permanence (b) (*F* value = 41.6) of the animals in the open arms of the elevated plus maze, (c) number of entries in closed arms (*F* value = 21.2), and (d) time of length of stay in closed arms (*F* value = 20.7). The column represents the average ± S.E.M. (*n* = 8). Statistical analysis: ANOVA unidirectional followed by the Tukey test, ^∗^*p* < 0.05, ^∗∗^*p* < 0.01, ^∗∗∗∗^*p* < 0.001: (HC) = vs.control and (DZP) = vs.control.

**Figure 3:** Effect of HC (mg/kg, i.p.), number of crossings (a) (*F* value = 15.9), number of rearing (b) (*F* value = 20.5), and number of grooming (c) (*F* value = 13.6), on open field test. The column represents the average ± S.E.M. (*n* = 8). Statistical analysis: ANOVA unidirectional followed by the Tukey test, ^∗^*p* < 0.05, ^∗∗^*p* < 0.01, ^∗∗∗∗^*p* < 0.001: (HC) = vs.control and (DZP) = vs.control.

**Figure 4:** Influenced the HC after using flumazenil in the number of entries (a) (*F* value = 59.2) and the time permanence (b) (*F* value = 56.3) of animals in EPM. The column represents the average ± S.E.M. (*n* = 8). Statistical analysis: ANOVA unidirectional followed by the Tukey test, ^∗^*p* < 0.05, ^∗∗^*p* < 0.01, ^∗∗∗∗^*p* < 0.001: (HC) = vs.control and (DZP) = vs.control.

**Figure 5:** Visualization of interactions 2D and 3D between the binders HC and ABU and the target GABA_A_. Complex GABA_A_-HC (a). 3D and 2D interactions between the ligand HC and GABA_A_ amino acids (b, c). 3D and 2D interactions between the ABU ligand and amino acids GABA_A_ (d, e). In green, the interactions of hydrogens are represented; in orange, electrostatic interactions; in red, steric interactions; and in purple, hydrophobic interactions.

**Figure 6:** Values of the molecular dynamics. (a) RMSD of C*α* atoms of GABA_A_R isolated and complexed with HC and ABU ligands. (b) RMSD of the C*α* atoms of the HC and ABU ligands. (c) RMSF of C*α* atoms of GABA_A_R complexed with HC and ABU ligands.

**Figure 7:** Molecular dynamics simulation during 1000 ps. Structure of the GABA_A_R-HC complex and its active site (a), initial structure (b), 200 ps (c), 400 ps (d), 600 ps (e), 800 ps (f), and 1000 ps (g).

**Table 1:** Results of the binding energy values (kcal/mol) in five different scoring functions.

Molecule	Moldock (MVD)	Goldscore (Gold)	Binding energy (AutoDock Vina)	Binding energy (AutoDock)	Chempl (Plants)
Gamma-aminobutyric acid (GABA_A_)					
HC	-75.40	29.52	-4.8	-5.38	37.94
PDB ABU	-88.65	26.22	-5.7	-4.95	20.96

**Table 2:** *In silico* pharmacokinetic data estimated using SwissADME or pkCSM web services.

Compound	Log*P*^a^	Log*S*^b^	TPSA (Å^2^)^c^	Caco-2 permeability (log Papp; log cm/s)^d^	Int. Abs. (%)^e^	VDss (log L/kg)^f^	Fract. Unb.^g^	Total clearance (log mL/min/kg)^h^
HC	2.15	-2.04	37.30	1.49	93.84	-0.04	0.50	1.36

^a^SwissADME Moriguchi log of octanol-water partition coefficient. ^b^SwissADME Ali log of aqueous solubility. ^c^SwissADME calculation of Topological Polar Surface Area (TPSA). ^d^pkCSM prediction of Caco-2 cell permeability as estimation of absorption in human intestinal mucosa. ^e^pkCSM prediction of the proportion of compound absorption thought the human small intestine.^f^pkCSM prediction of the log of steady state volume of distribution (VDss). ^g^pkCSM prediction of compound fraction unbound in plasma (not bound to serum proteins). ^h^pkCSM prediction of the log of total drug clearance.

## Data Availability

Some or all data, models, or code generated or used during the study are available from the corresponding author by request.
